The article "Boosted Sine Cosine Algorithm with Application to Medical Diagnosis" was published in 2022. Journal: Comput Math Methods Med.

# Boosted Sine Cosine Algorithm with Application to Medical Diagnosis

**DOI:** 10.1155/2022/6215574

**Published:** 2022-06-22

**Authors:** Xiaojia Ye, Zhennao Cai, Chenglang Lu, Huiling Chen, Zhifang Pan

**Affiliations:** ^1^Shanghai Lixin University of Accounting and Finance, Shanghai 201209, China; ^2^College of Computer Science and Artificial Intelligence, Wenzhou University, Wenzhou 325035, China; ^3^College of Modern Information Technology, Zhejiang Institute of Mechanical and Electrical Engineering, Hangzhou, Zhejiang 310051, China; ^4^The First Affiliated Hospital of Wenzhou Medical University, Wenzhou 325000, China

## Abstract

The sine cosine algorithm (SCA) was proposed for solving optimization tasks, of which the way to obtain the optimal solution is mainly through the continuous iteration of the sine and cosine update formulas. However, SCA also faces low population diversity and stagnation of locally optimal solutions. Hence, we try to eliminate these problems by proposing an enhanced version of SCA, named ESCA_PSO. ESCA_PSO is proposed based on hybrid SCA and particle swarm optimization (PSO) by incorporating multiple mutation strategies into the original SCA_PSO. To validate the effect of ESCA_PSO in handling global optimization problems, ESCA_PSO was compared with quality algorithms on various types of benchmark functions. In addition, the proposed ESCA_PSO was employed to tune the best parameters of support vector machines for dealing with medical diagnosis tasks. The results prove the efficiency of the proposed algorithms in solving optimization problems.

## 1. Introduction

### 1.1. Motivation

Many problems in real life can be summarized as global optimization problems. When it comes to increasingly complex optimization problems, traditional methods are generally unsatisfactory [1]. Therefore, many scholars began to explore new solutions. The metaheuristic algorithm (MA) is developed for obtaining and grasping information to effectively find approximately optimal solutions through learning strategies. MA has been applied to many scenarios owing to its effective optimization capability [2]. For example, MA has found the great potential in wind speed prediction [3], scheduling problem [4], parameter optimization [5], PID optimization control [6], gate resource allocation [7], fault diagnosis of rolling bearings [8], cloud workflow scheduling [9], energy vehicle dispatch [10], combination optimization problems [11], traveling salesman problem [12], object tracking [13], neural network training [14], and multiattribute decision making [15].

In 2016, a new swarm intelligence algorithm named sine cosine algorithm (SCA) [16] was proposed. SCA searches the solution based on the sine function and cosine function. It owns strong global searchability, which can significantly increase the global optimal solution through enough iterations. However, SCA also is faced with some problems, for instance, slow convergence speed, low convergence accuracy, and easily falling into local optimum. To overcome the problems existing in SCA, a hybrid SCA and PSO algorithm (SCA_PSO) was put forward by Nenavath et al. [17], which aims to solve optimization problems and target tracking. The search mechanism of the PSO algorithm is added to the traditional SCA to guide the search for potential candidate solutions. It should be noted that though the SCA_PSO has achieved promising results on object tracking when dealing with complex problems, it is still easy to skip the true optimal solution and lead to premature convergence.

The article "Boosted Sine Cosine Algorithm with Application to Medical Diagnosis" was published in 2022. Journal: Comput Math Methods Med.

According to “No Free Lunch” [18], we have introduced the differential evolution algorithm (DE) and combined mutation strategies into the original SCA_PSO to strengthen its capability of local search and reduce the occurrence of premature convergence. The proposed ESCA_PSO was validated on a benchmark test which includes various types of functions. Experimental results demonstrated that ESCA_PSO was significantly better than SCA_PSO and other competitive counterparts. In addition, the ESCA_PSO was also used to construct an optimal support vector machine model (SVM) to deal with the medical diagnosis problems in an effective manner. In general, ESCA_PSO has improved the performance of SCA_PSO in a significant manner.

### 1.2. Literature Review

SCA has been widely studied and applied in many fields because of its simple implementation and relatively excellent performance in realizing complex problems. For example, SCA was employed to tackle the scheduling problem in [19]. A multiobjective SCA was proposed to solve engineering optimization problems in [20] and forecast the wind speed in [21]. SCA was employed to predict the time series by constructing an optimal support vector regression model in [22]. In [23], SCA was utilized to optimize the parameters of fuzzy *k*-nearest neighbor to build an optimized classifier for predicting the intention of students for a postgraduate entrance examination. In [24], SCA was applied to optimize the SVM's parameters and the boosted classifier was trained to predict students' entrepreneurial intentions.

In addition to applications, scholars have also proposed many improved SCA variants. Issa et al. [25] proposed a new idea of SCA, that is, the combination of SCA and PSO. This algorithm was used to solve the problem of pairwise local alignment to look for the longest continuous substring between two biological sequences, which has shown good performance in accuracy and calculation time. Nenavath and Jatoth [26] proposed to select the DE algorithm to merge into SCA and applied it to target tracking. Abd Elaziz et al. [27] mutated SCA (OBSCA) with opposition-based learning mechanisms, which has effectively boosted SCA's search efficiency and expanded its search scope. Qu et al. [28] improved the SCA by adding three strategies. Kumar et al. [29] tried to mix SCA with Cauchy and Gaussian distributions, which were named CGSCA. Simulations showed that the single-sensor tracking scheme based on CGSCA had better results in terms of tracking time and tracking efficiency. Long et al. [30] combined SCA with inertia weight based on a position updating equation and a nonlinear conversion parameter strategy to ameliorate SCA's ability in solving high-dimensional problems. Tu et al. [24] proposed to adopt the chaotic local search enhanced SCA for training an optimal support vector machine to predict students' entrepreneurial intentions. Turgut [31] proposed that mixing SCA with a backtracking search algorithm (BSA) was an efficient way to realize the shell and tube evaporator's optimal design. With the proposed optimization method, the optimal values of the total design cost of the heat exchanger and the total heat transfer coefficient were better than the results of the other optimizers in the literature. Guo et al. [32] introduced the Riesz fractional derivative and the OBL strategy into SCA and applied the method to deal with the engineering problems. Gupta and Deep [33] proposed to add a leading guidance mechanism and simulated quenching algorithm together to SCA and applied it to train multilayer perceptron. Gupta and Deep [34] utilized the OBL strategy and the self-adaptive component to enhance the SCA. And this improved algorithm's efficacy was confirmed by lots of benchmark problems and engineering problems. Tawhid and Savsani [20] proposed a novel and effective multiobjective version of SCA (MO-SCA). The difference between MO-SCA and SCA is mainly reflected in two aspects, one is to improve the nondominated level by adding an elite nondominated sorting strategy, and the other is to maintain the diversity of optimal solutions by adding crowded distance method. At present, machine learning methods are still a research hotspot [35–42]. However, the hyperparameters of the model have a crucial impact on its performance. Therefore, combining the improved version of SCA with machine learning methods to obtain the best hyperparameter combination model is also a novel research angle.

The article "Boosted Sine Cosine Algorithm with Application to Medical Diagnosis" was published in 2022. Journal: Comput Math Methods Med.

### 1.3. Contribution and Paper Organization

The main contributions of this study are as follows:

- An improved SCA named ESCA_PSO is proposed
- The proposed ESCA_PSO has achieved superior performance to other peers on function optimization and machine learning tasks
- Successfully applied ESCA_PSO to SVM parameter optimization problem
- Successfully use ESCA_PSO-SVM in the field of medical diagnosis

The rest part of this paper is assigned as follows: The introduction of SCA and SCA-PSO is arranged in Section 2. Our proposed ESCA_PSO is presented in Section 3. The details information on experimental results and discussions are described in Section 4. Finally, in Section 5, conclusions and future works are summarized.

## 2. An Overview of SCA_PSO Algorithm

### 2.1. Standard SCA

In recent years, many new intelligent algorithms have been proposed to solve practical problems, such as hunger games search (HGS) [43], weighted mean of vectors (INFO) [44], Harris hawks optimization (HHO) [45], slime mould algorithm (SMA) [46], and Runge Kutta optimizer (RUN) [47]. These algorithms have shown great potential in various fields such as engineering, medicine, energy, finance, and education. In 2016, Mirjalili [16] put forward a novel swarm intelligence algorithm called SCA for global optimization tasks. Similar to other metaheuristics, it looks for the solution in a random searching space. SCA obtains the optimal solution through triangle sine cosine functions [16].

The following location updating formulas are proposed for two phases:

(1) $$\begin{array}{c} X_{i}^{t+1}=X_{i}^{t}+r_{1}\times \sin\left(r_{2}\right)\times \left|r_{3}P_{i}^{t}-X_{i}^{t}\right|, \end{array}$$

(2) $$\begin{array}{c} X_{i}^{t+1}=X_{i}^{t}+r_{1}\times \cos\left(r_{2}\right)\times \left|r_{3}P_{i}^{t}-X_{i}^{t}\right|, \end{array}$$

where *X*_*i*_^*t*^ is the position of the current solution in *i*-th dimension at *t*-th iteration,  *r*_1_,*r*_2_, *r*_3_ are random numbers, *P*_*i*_ is the position of the target point in *i*-th dimension, and || indicates absolute value.

Combining the above, the following equation can be obtained:

(3) $$\begin{array}{c} X_{i}^{t+1}=\left\{\begin{array}{c} X_{i}^{t}+r_{1}\times \sin\left(r_{2}\right)\times \left|r_{3}P_{i}^{t}-X_{i}^{t}\right|,r_{4}<0.5,\\ X_{i}^{t}+r_{1}\times \cos\left(r_{2}\right)\times \left|r_{3}P_{i}^{t}-X_{i}^{t}\right|,r_{4}\geq 0.5, \end{array}\right. \end{array}$$

where *r*_4_ is a random number in the range [0, 1].

As the above formulae reveal, *r*_1_, *r*_2_, *r*_3_ and *r*_4_ are four important parameters with different meanings. The *r*_1_ mainly decides whether the position of the next move is within the boundary range of solution and destination or outside the range. *r*_2_ represents the distance required for the movement to reach the destination. The coefficient *r*_3_ carries a random load for the destination to stochastically emphasize (*r*_3_> 1) or deemphasize (*r*_3_ <1) the effect of destination in describing the distance. *r*_4_ switches from sine function to cosine function or vice versa in Eq. (3). The values of *r*_2_ were set in [0, 2*π*]  in this study.

The article "Boosted Sine Cosine Algorithm with Application to Medical Diagnosis" was published in 2022. Journal: Comput Math Methods Med.

To achieve a steady global and local search, the range of sine and cosine functions in Eqs. (1)–(3) are altered adaptively according to the following formula:

(4) $$\begin{array}{c} r_{1}=a-t\frac{a}{T}, \end{array}$$

where *t* means the current iteration, *T* means the maximum number of iterations, and *a* is a constant with the value of 2.

### 2.2. SCA_PSO Algorithm

To eliminate the shortcoming of SCA, Nenavath et al. [17] came up with an improved hybrid SCA_PSO for dealing with optimization tasks. The SCA_PSO integrates PSO's strengths in exploitation and the SCA's strengths in exploration to approach the global optimal solution.

By adding internal storage to SCA, each individual is permitted to follow the coordinates associated with the adaptive values in the search space. And the personal historical best solution of each search agent in the present population is stored in the form of a matrix, SCA-*P*_best_, which is the same as the concept of *P*_best_ in PSO each iteration. In addition, the solution also keeps track of the optimal value achieved so far by any nearby solution. As a new concept in SCA, *P*_best_ and *G*_best_ enhance the exploitation ability of SCA. The pseudocode of SCA_PSO is shown in Pseudocode 1.

## 3. Proposed ESCA_PSO

The improved ESCA_PSO is combined with two efficient strategies. Firstly, a DE with the “random variation” mode is successfully combined with the SCA_PSO to strengthen the global search capability of the SCA_PSO. Then, a combined mutation with the mixed distributions of Gaussian, Cauchy, and Lévy was added to the combination mutation strategy, which can further improve the accuracy of the solution.

### 3.1. Combined Mutation of Gaussian, Cauchy, and Lévy

Gaussian distribution (GD) [48] is a significant probability distribution in many subjects such as engineering and mathematics. GD has many excellent features. Plenty of random variables and objects in nature can be presumably expressed as GD, and many probability distributions can be approximated or exported by this distribution. The probability density function of the GD can be expressed according to Eq. (5):

(5) $$\begin{array}{c} f\left(x\right)=\frac{1}{\sqrt{2\pi }\sigma }\exp\left(-\frac{{\left(x-\mu \right)}^{2}}{2\sigma^{2}}\right), \end{array}$$

where *μ* and *σ* represent the mean and standard deviation, respectively.

The article "Boosted Sine Cosine Algorithm with Application to Medical Diagnosis" was published in 2022. Journal: Comput Math Methods Med.

Cauchy distribution [49] is also called Cauchy-Lorentz distribution. It is a continuous probability distribution named after Augustine-Louis-Cauchy and Hendrick-Lorentz. It is similar to normal distribution. Cauchy distribution is also widely used in statistics. It has the characteristics of the nonexistence of expectation and variance and additivity. The probability density function of the Cauchy distribution can be expressed according to Eq. (6):

(6) $$\begin{array}{c} f\left(x;x_{0},y\right)=\frac{1}{\pi }\left(\frac{\gamma }{{\left(x-x_{0}\right)}^{2}+\gamma^{2}}\right), \end{array}$$

where *x*_0_ is the position parameter defining the location of the distribution peak; *γ* is the scale parameter defining half the width of the maximum half.

Lévy flights [50] based on Lévy distribution are consistent with the search behavior of many organisms in the nature and are widely used in optimization algorithms and optimal search processes. Moreover, the stochastic process can maximize the search efficiency of resources under uncertain conditions. In the search process, Lévy flights can make the whole search process more effective and stable, balancing the proportion of local search and global search. Due to the existence of the random process of the Lévy flight, the short-range exploratory local search and the occasional long-distance walk are in phase. Thus, the algorithm's local searching speed is faster, and the solutions are more easily searched near the current optimum. The decomposition can search far away from the current optimal value, thus ensuring that the algorithm does not fall into the local optimum (LO). The Lévy formula used is as follows:

(7) $$\begin{array}{c} \sigma ={\left(\frac{\Gamma \left(1+\beta \right)\sin\left(\pi \beta /2\right)}{\Gamma \left[1+\beta /2\right]\beta 2^{\beta ‐1/2}}\right)}^{\left(1/\beta \right)}, \end{array}$$

where *Γ* (*x*) is a continuation function of the factorial, that is, when the *x* is a positive integer Γ(*x* + 1) = *x*! The value of the variable *β* determines the shape of the Lévy probability density function, especially in the tail area.

(8) $$\begin{array}{c} \gamma =\frac{\mu }{{\left|v\right|}^{1/\beta }}, \end{array}$$

where *γ* is the flight step, *v*, is the standard normal distribution, and *μ* is a normal distribution with the mean of 0 and the variance of *σ*^2^.

### 3.2. Combined Mutation Strategy

As mentioned in the foregoing, the DE algorithm can enhance the global search capability of SCA_PSO, while mutation of Gaussian, Cauchy, and Lévy is algorithms that can make the algorithm perform better in local search. A combined mutation strategy was proposed in this study, which combined the different characteristics of the three mutation strategies, making the SCA_PSO find a more balanced manner in performing explorative search and exploitative search. The whole algorithm steps are as shown below:

Step 1. Search using the mentioned SCA.

The article "Boosted Sine Cosine Algorithm with Application to Medical Diagnosis" was published in 2022. Journal: Comput Math Methods Med.

Step 2. Mutate the SCA_PSO by the DE algorithm and the new individual will be retained if its fitness value is better than the original one.

Step 3. Update using the formula of SCA_PSO. The update formula used is as follows:

(9) $$\begin{array}{c} v\left(k\right)=w∙v\left(k\right)+c1∙r2∙\left(p\text{best}-x_{i}^{k}\right)+c2∙r3∙\left(SCA_{{G_{\text{best}}}_{x_{i}^{k}}}\right), \end{array}$$

(10) $$\begin{array}{c} x_{i}^{k}=x_{i}^{k}+v\left(k\right), \end{array}$$

where *c*1,  *c*2=2. *r*2, and  *r*3 are in the range of [0, 1].

Step 4. Use combined mutation of Gaussian, Cauchy, and Lévy to mutate the current optimal individuals, find the individuals with the smallest of the three results, and update the fitness values and corresponding individuals.

(11) $$\begin{array}{c} X=\min\left\{\left.X\_m\_\text{Levy},X\_m\_\text{gaus},X\_m\_\text{cauchy}\right\}\right., \end{array}$$

(12) $$\begin{array}{c} X_{m_{\text{gaus}}}=X_{i}^{t}∙\left(1+k∙\text{randn}\right), \end{array}$$

(13) $$\begin{array}{c} X_{m_{\text{cauchy}}}=X_{i}^{t}∙\left(1+k∙\text{cauchy}\right), \end{array}$$

(14) $$\begin{array}{c} X_{m_{\text{Levy}}}=X_{i}^{t}∙\left(1+k∙\text{Levy}\left(1\right)\right), \end{array}$$

where *X_m_*Lévy, *X_m_*gaus, and *X_m_*cauchy are the values obtained by the Lévy, Gaussian, and Cauchy strategies, respectively.

Pseudocode 2 and Figure 1 display the detailed steps and flowchart of ESCA_PSO, respectively.

First of all, the current optimal individual *SCA*_*G*_best_ is obtained by SCA. Then, the particle swarm population is initialized with the help of *SCA*_*G*_best_ and mutated with the help of DE strategy. Next, the population is updated using SCA_PSO. Finally, it is updated by Gaussian, Cauchy, and Lévy flight strategies.

### 3.3. Complexity Analysis

The time complexity of the ESCA_PSO is mainly related to the number of four factors, which are algorithm iterations (*T*), PSO's iterations (*P*), population (*N*), and dimensions (*D*). And the whole time complexity is analyzed as follows: *O* (ESCA_PSO) = *O* (initialize) + *T* × (*O* (calculate the fitness of population) + *O* (update location with SCA) + *P* × (*O* (calculate the fitness of population) + *O* (update location with PSO)) + *O* (perform combined mutation strategy)). The time complexity of initialization is *O*(*N* × *D*). Since there are *N* individuals, the fitness of the initial populations is *O* (*N*). Updating location with SCA is *O* (*N*). Updating location with PSO is *O* (*N* × *D*). Performing the combined mutation strategy is *O* (*N*). All in all, it is not difficult to conclude that the total time complexity of ESCA_PSO is *O* (ESCA_PSO) = *O* (*N* × *D*) + *T* × (*O* (*N*) + O (*N*) + *P* × (O (*N*) + O (*N* × *D*)) + O (*N*)) = O (*N* × *D*) + *T* × (2O (*N*) + *P* × (O (*N*) + O (*N* × *D*)) + O (*N*)).

The article "Boosted Sine Cosine Algorithm with Application to Medical Diagnosis" was published in 2022. Journal: Comput Math Methods Med.

## 4. Experimental Results

To confirm the effectiveness of ESCA_PSO, the proposed ESCA_PSO is compared with other competitive metaheuristic algorithms on 30 functions of CEC2014 in this part. And then ESCA_PSO carries on the variation mechanism contrast experiment. Finally, ESCA_PSO is used for tuning SVM's parameters for medical diagnosis purposes.

### 4.1. Benchmark Functions

This experiment used 30 classical functions to substantiate the proposed method and other competitors. These functions include unimodal, multimodal, composition, and hybrid functions. F1-F3 are unimodal functions, F4-F16 are multimodal functions, and F17-F22 are hybrid functions. F23-F30 are composition functions, which are selected from CEC2014. These 30 different benchmark functions can comprehensively estimate the performance of the ESCA_PSO. The related descriptions are demonstrated in Table 1, where range means the boundary of the search space for the relevant functions. As we all know, a unimodal function corresponds to a globally optimal solution; so, it can be employed to benchmark development capability. Conversely, the multimodal function possesses a lot of LO solutions, which leads to the algorithm falling into LO. Such functions can test the capability of the method to refrain from stagnation and exploration ability. Moreover, both the hybrid function and multimodal function only have one global optimum but multiple LO solutions. The structures of composition functions are more complex.

All the algorithms in the following experiments are coded on MATLAB 2014b. And to be fair, the experimental verification is carried out under the unified condition, i.e., the population size is set to 30, the maximum evaluation time is set to 300000, the dimension is set to 30, and the number of runs is set to 30.

### 4.2. Comparison with Other Algorithms

In this experiment, the ESCA_PSO was contrasted to SCA, GWO [51], MFO [52], BA [53], and PSO [54] on the functions presented in Table 1. To further validate the effect of the proposed ESCA_PSO, two improved SCA variants including SCA_PSO and SCADE [26] were involved for comparison and compare with LSHADE [55] which is the champion algorithm of CEC2014. The parameter configuration of algorithms is shown in Table 2. The detailed comparison results including the average value (Avg) of the best solution and standard deviation (Std) of every approach in 30 independent runs are displayed in Table 3.

The article "Boosted Sine Cosine Algorithm with Application to Medical Diagnosis" was published in 2022. Journal: Comput Math Methods Med.

We can see that the advantages of ESCA_PSO are not very obvious in the unimodal functions and multimodal functions. In these functions, ESCA_PSO is slightly better than the original algorithm SCA and its variants CGSCA and SCADE. But compared with high-quality algorithms such as LSHADE, there is still a certain gap. However, ESCA_PSO has a very good performance in the complex structure of the composition functions. Compared with other algorithms on F23-F30, it ranks first or second.

By the Friedman test, we can get the average ranking of test algorithms, which is usually used to get the difference between many test results. At the same time, to further analyze the experimental structure, Wilcoxon signed-rank test was adopted for statistical work.

In Table 4, all experimental results were taken from those two tests mentioned above. AVG in the table represents the average ranking of algorithms obtained by the Friedman test, and “+/-/=” represents the performance of the function compared with ESCA_PSO. Specifically, “+” means ESCA_PSO is better than this algorithm, “-” indicates that ESCA_PSO is inferior to this algorithm, and “=” means that the performance is similar to ESCA_PSO. In Wilcoxon signed-rank test, when the *p* value is less than 0.05, the performance between the two algorithms is significant. It was also used to evaluate the significance of ESCA_PSO versus other approaches. It can see from the table that ESCA ranks second on average, which is better than other algorithms overall. Compared with SCA, SCADE, CGSCA, GWO, and MFO, it is significantly better than 20 functions. However, it is indeed weaker than the champion algorithm LSHADE on multimodal functions and unimodal functions.

Figure 2 shows nine graphs of convergence we selected. As shown in Figure 2, it can be seen that ESCA_PSO does have a good convergence rate on these functions. It quickly converges to a lower point. And ESCA_PSO has a significant improvement over than original SCA. Of course, it is undeniable that some algorithms converge faster than ESCA_PSO, but ESCA_PSO has higher quality solutions.

Despite the great potential of the proposed ESCA_PSO, the approach of sacrificing a certain time complexity in exchange for an increase in terms of accuracy is insufficient side. Nevertheless, the algorithm is still competitive with LSHADE in unimodal and multimodal functions.

### 4.3. Comparison of Mutation Mechanism

As mentioned earlier, three mutation mechanisms were added to ESCA_PSO. To further analyze ESCA_PSO, we conducted comparative experiments on the mutation mechanism of ESCA in this section.

The article "Boosted Sine Cosine Algorithm with Application to Medical Diagnosis" was published in 2022. Journal: Comput Math Methods Med.

To compare the mutation mechanism, we construct three algorithms, namely, ESCA_PSO1, ESCA_PSO2, and ESCA_PSO3. Compared with ESCA_PSO, ESCA_PSO1 only uses Gaussian mutation while others remain unchanged. By analogy, ESCA_PSO2 only uses the Cauchy mutation while ESCA_PSO3 only uses the Lévy mutation. The population dimension and the total number of iterations of this experiment are the same as those in the previous experiment settings.

The results obtained from the experiments are shown in Table 5, and there is not much difference between these four algorithms, which can be concluded by comparing the whole data. This is because most of the four algorithms are the same, and only the mutation mechanism has changed. From the numerical value obtained from the experiment, ESCA_PSO has not achieved the best results in functions many times. But relatively, ESCA_PSO is rarely ranked last. This is also because ESCA_PSO integrates three mutation mechanisms, which makes it applicable to more functions.

Figure 3 shows several convergence graphs in this experiment. From the figure, we can see that in F2, F17, and F19, the convergence curves of the four algorithms are relatively similar, and there is no big difference in general. In F27 and F28, the performance of ESCA_PSO3 is not as good as the other three algorithms. In F29 and F30, ESCA_PSO2 is quite different from the other three algorithms. However, ESCA_PSO can keep a good level in these functions. This shows that the combination of three different mutation mechanisms can help the algorithm adapt to more functions.

However, ESCA_PSO that we proposed is not perfect, and there are certain limitations. In the benchmark functions experiment, it can be seen that there is still a gap between the performance of this algorithm and champion algorithms in unimodal functions and multimodal functions.

### 4.4. ESCA_PSO For Optimization of SVM

Like many other machine learning methods [56], SVM has many advantages such as “simple structure,” “overcoming dimension disaster,” and “small sample,” which can overcome the weaknesses of conventional neural networks such as poor learning and generalization ability [57]. Since its introduction, SVM has found its application in many practical problems. Practice shows that the penalty factor *C* and kernel function variable *g* have the key influence on the recognition accuracy of the SVM model when solving the recognition problem based on the radial basis kernel function. When the penalty factor *C* is small, the recognition rate of training and test samples is low, and the SVM is under learning. When *C* is too large, the accuracy of the training sample is higher, the test sample recognition rate is lower, and the SVM is overlearning. The smaller the kernel function parameter *g* is, the higher the training sample recognition rate is and the lower the accuracy of the test sample is. When *g* is larger, the accuracy of training and test samples becomes lower, and SVM is under learning. Traditional methods such as trial and error method and network search method cannot meet the requirements of accuracy in practical application. Currently, with the development and maturity of MAs, good results have been achieved in improving the performance of the SVM model. For example, Li et al. [58] proposed moth-flame optimization (MFO) to tune the best parameters of SVM and applied it to the diagnosis of tuberculous pleural effusion. Li et al. [59] proposed a chaotic enhanced gravitational search algorithm (GSA) for optimizing the parameters of SVM. Das et al. [60] proposed to use the teaching-learning-based optimization (TLBO) for parameter optimization of SVM, and the good performance was validated by a financial case. Tang et al. [61] proposed a Lévy flight-based shuffled frog-leaping algorithm for determining the best parameters of SVM. Ahmadi et al. [62] developed the imperialist competition algorithm (ICA) to determine the best parameters of SVM for stock market timing. Li et al. [22] proposed SCA to tune the best parameters of SVM, and the good results were verified on several benchmark datasets. Rojas-Dominguez et al. [63] proposed to use several metaheuristics to search for the best parameters of SVM, and the results showed that the estimation of distribution algorithms can achieve the best results. Tharwat et al. [64] proposed a chaotic antlion optimizer for tuning the best parameters, and the effectiveness was validated on an array of well-known datasets. Bablani et al. [65] proposed to use the bat algorithm (BA) to simultaneously determine the optimal parameters of SVM and the best subset of features and applied the model for dealing with the electroencephalography (EEG) data.

The article "Boosted Sine Cosine Algorithm with Application to Medical Diagnosis" was published in 2022. Journal: Comput Math Methods Med.

In this study, we applied ESCA_PSO to search for the best parameters of SVM, and the resultant model was called ESCA_PSO-SVM as shown in Figure 4. ESCA_PSO-SVM was applied to predict two different medical problems including the Bupa liver and the Cleveland heart.

The Bupa liver diabetes dataset has a total of 345 samples and 7 features.  Table 6 demonstrates the detailed results got by ESCA_PSO-SVM via 10-fold crossvalidation. As shown in Table 6, ESCA_PSO-SVM has got an average accuracy (ACC) of 73.04%, an average sensitivity of 59.18%, an average specificity of 83.81%, and an average Mathews correlation coefficient (MCC) of 0.4404.

From Figure 5, it is clear that ESCA_PSO-SVM has more excellent performance than SCA-SVM in such four indexes. Moreover, compared with the prediction accuracy, the ESCA_PSO-SVM has the best precision, while the KNN model has the lowest precision. Based on the sensitivity metric, ESCA_PSO-SVM ranked second, while BP obtained the worst values. In terms of the obtained specificity, ESCA_PSO-SVM was the best, followed by SVM, SCA-SVM, BP, KNN, and CART. In terms of the MCC, ESCA_PSO-SVM provided the best value, followed by SVM, SCA-SVM, CART, BP, and KNN. It suggests that ESCA_PSO-SVM is more advantageous and stable in solving the Bupa liver problem.

The Cleveland heart data was got from the UCI repository, and it includes 303 samples and 76 features.  Table 7 shows the detailed results of ESCA_PSO-SVM through 10-fold crossvalidation on this dataset. From Table 7, ESCA_PSO-SVM has got an average ACC of 82.81%, a sensitivity of 76.88%, a specificity of 86.38%, and an MCC of 0.6486.

In Figure 6, ESCA_PSO-SVM is superior to SCA-SVM in terms of four evaluation indexes. Concerning the classification accuracy, it can be seen clearly that the ESCA_PSO-SVM has got the best ACC, whereas BP has the lowest precision. In terms of the sensitivity metric, the value of SVM is the same as that of ESCA_PSO-SVM which takes the first place. As for the specificity metric, although SCA-SVM ranked first place, it was only slightly superior to ESCA_PSO-SVM. According to the MCC metric, ESCA_PSO provided the best value, followed successively by SCA-SVM, SVM, KNN, CART, and BP. These all proved the robustness and stableness of the ESCA_PSO-SVM on the Cleveland heart problem. Shortly, many problems are waiting to be optimized for which ESCA_PSO can be applied, such as disease module identification [66], molecular signatures identification for cancer diagnosis [67], drug-disease associations prediction [68], drug discovery [69], and pharmacoinformatic data mining [70].

## 5. Conclusions and Future Directions

To make up for the deficiency of SCA_PSO, this paper proposed ESCA_PSO, an enhanced version of SCA_PSO. The chance of prematurely falling into convergence was effectively reduced by introducing DE and joint mutation mechanisms. To verify its performance, it was compared with seven advanced algorithms on 30 benchmark function sets. The experimental results showed that the performance of the proposed algorithm was better than that of the traditional optimization algorithms and had certain competitiveness with LSHADE. Inspired by the “No Free Lunch” theory, this paper further explored the application of ESCA_PSO in medical diagnosis and successfully applied it to hyperparameter optimization of support vector machine.

The article "Boosted Sine Cosine Algorithm with Application to Medical Diagnosis" was published in 2022. Journal: Comput Math Methods Med.

The results showed that the support vector machine model combined with the proposed algorithm outperformed the other five existing models and achieved an average accuracy of 82.81%. In conclusion, the proposed algorithm can be regarded as a reliable technique for solving practical problems.

For future work, there are still many problems worthy of study. First of all, we will continue to improve the algorithm, by means such as trying to introduce other metaheuristic algorithms or optimizing the time complexity while ensuring the effect. In addition, we will try to apply ESCA_PSO to other fields such as image segmentation, clustering optimization, and discrete optimization.

## Figures and Tables

**Figure 1:** Flowchart of ESCA_PSO.

**Figure 2:** Convergence curves of ESCA_PSO and other algorithms 9 selected benchmark functions.

**Figure 3:** Convergence curves of ESCA_PSO and other algorithms 9 selected benchmark functions.

**Figure 4:** Flowchart of ESCA_PSO-SVM.

**Figure 5:** Comparison between the ESCA_PSO-SVM and other methods on the Bupa liver problem.

**Figure 6:** Comparison between the ESCA_PSO-SVM and other methods on the Cleveland heart problem.

**Pseudocode 1:** The pseudocode of the SCA_PSO.

**Pseudocode 2:** Pseudocode of the ESCA_PSO.

**Table 1:** Description of 30 benchmark functions.

ID	Function equation	Range	Optimum value
Unimodal functions			
F1	Rotated high conditioned elliptic function	[-100, 100]	*f*_1_{*X*_min_} = 100
F2	Rotated bent cigar function	[-100, 100]	*f*_2_{*X*_min_} = 200
F3	Rotated discus function	[-100, 100]	*f*_3_{*X*_min_} = 300
Simple multimodal functions			
F4	Shifted and rotated Rosenbrock's function	[-100, 100]	*f*_4_{*X*_min_} = 400
F5	Shifted and rotated Ackley's function	[-100, 100]	*f*_5_{*X*_min_} = 500
F6	Shifted and rotated Weierstrass function	[-100, 100]]	*f*_6_{*X*_min_} = 600
F7	Shifted and rotated Griewank's function	[-100, 100]	*f*_7_{*X*_min_} = 700
F8	Shifted Rastrigin's function	[-100, 100]	*f*_8_{*X*_min_} = 800
F9	Shifted and rotated Rastrigin's function	[-100, 100]	*f*_9_{*X*_min_} = 900
F10	Shifted Schwefel's function	[-100, 100]	*f*_10_{*X*_min_} = 1000
F11	Shifted and rotated Schwefel's function	[-100, 100]	*f*_11_{*X*_min_} = 1100
F12	Shifted and rotated Katsuura function	[-100, 100]	*f*_12_{*X*_min_} = 1200
F13	Shifted and rotated HappyCat function	[-100, 100]	*f*_13_{*X*_min_} = 1300
F14	Shifted and rotated HGBat function	[-100, 100]	*f*_14_{*X*_min_} = 1400
F15	Shifted and rotated expanded Griewank's plus Rosenbrock's function	[-100, 100]	*f*_15_{*X*_min_} = 1500
F16	Shifted and rotated expanded Scaffer's F6 function	[-100, 100]	*f*_16_{*X*_min_} = 1600
Hybrid functions			
F17	Hybrid function 1 (*N* = 3)	[-100, 100]	*f*_15_{*X*_min_} = 1700
F18	Hybrid function 2 (*N* = 3)	[-100, 100]	*f*_16_{*X*_min_} = 1800
F19	Hybrid function 3 (*N* = 4)	[-100, 100]	*f*_17_{*X*_min_} = 1900
F20	Hybrid function 4 (*N* = 4)	[-100, 100]	*f*_18_{*X*_min_} = 2000
F21	Hybrid function 5 (*N* = 5)	[-100, 100]	*f*_19_{*X*_min_} = 2100
F22	Hybrid function 6 (*N* = 5)	[-100, 100]	*f*_22_{*X*_min_} = 2200
Composition functions			
F23	Composition function 1 (*N* = 5)	[-100, 100]	*f*_23_{*X*_min_} = 2300
F24	Composition function 2 (*N* = 3)	[-100, 100]	*f*_24_{*X*_min_} = 2400
F25	Composition function 3 (*N* = 3)	[-100, 100]	*f*_25_{*X*_min_} = 2500
F26	Composition function 4 (*N* = 5)	[-100, 100]	*f*_26_{*X*_min_} = 2600
F27	Composition function 5 (*N* = 5)	[-100, 100]	*f*_27_{*X*_min_} = 2700
F28	Composition function 6 (*N* = 5)	[-100, 100]	*f*_28_{*X*_min_} = 2800
F29	Composition function 7 (*N* = 3)	[-100, 100]	*f*_29_{*X*_min_} = 2900
F30	Composition function 8 (*N* = 3)	[-100, 100]	*f*_30_{*X*_min_} = 3000

The article "Boosted Sine Cosine Algorithm with Application to Medical Diagnosis" was published in 2022. Journal: Comput Math Methods Med.

**Table 2:** Parameters setting for involved algorithms.

Method	Parameter
ESCA_PSO	*a* = 2; *c*_1_ = 2; *c*_2_ = 2; *v*_max_ = 6
SCADE	cmin = 0.2; cmax = 0.8; pCR = 0.8
SCA	*a* = 2
SCA-PSO	*M* = 4; *N* = 9; vmax = 6; wmax = 0.9; wmin = 0.2
CGSCA	Delta = 0.1
GWO	*a* = [0, 2]
MFO	*b* = 1; *t* = [−1, 1]; *a* = [−1, −2]
BA	*a* = 0.5; *r* = 0.5
PSO	*c*_1_ = 2; *c*_2_ = 2; *v*_max_ = 6
LSHADE	Pb = 0.1; Ar = 1.4

**Table 3:** Results of ESCA_PSO versus other algorithms on 30 benchmark functions.

	F1		F2		F3	
	Avg	Std	Avg	Std	Avg	Std

ESCA_PSO	8.77*E*+06	3.47*E*+06	7.49*E*+07	7.38*E*+06	9.44*E*+03	2.27*E*+03
SCADE	4.23*E* +08	9.19*E*+07	2.97*E*+10	4.56*E*+09	5.46*E*+04	6.21*E*+03
SCA	2.52*E*+08	7.02*E*+07	1.76*E*+10	2.68*E*+09	3.72*E*+04	5.71*E*+03
SCA_PSO	8.01*E*+06	2.83*E*+06	3.83*E*+07	8.40*E*+06	2.99*E*+03	1.04*E*+03
CGSCA	2.85*E*+08	8.98*E*+07	1.82*E*+10	4.06*E*+09	4.15*E*+04	5.63*E*+03
GWO	5.76*E*+07	4.69*E*+07	2.18*E*+09	2.05*E*+09	3.24*E*+04	8.29*E*+03
MFO	8.50*E*+07	1.06*E*+08	1.22*E*+10	7.01*E*+09	1.10*E*+05	6.34*E*+04
BA	7.40*E*+05	2.88*E*+05	5.24*E*+05	2.80*E*+05	4.11*E*+02	1.40*E*+02
PSO	9.30*E*+06	2.45*E*+06	1.46*E*+08	1.63*E*+07	9.60*E*+02	9.65*E*+01
LSHADE	4.41*E*+03	7.34*E*+03	2.00*E*+02	3.77*E*-14	3.00*E*+02	1.74*E*-11

	F4		F5		F6	
	Avg	Std	Avg	Std	Avg	Std

ESCA_PSO	4.73*E*+02	3.72*E*+01	5.21*E*+02	4.33*E*-02	6.29*E*+02	3.45*E*+00
SCADE	2.40*E*+03	5.90*E*+02	5.21*E*+02	3.58*E*-02	6.35*E*+02	1.86*E*+00
SCA	1.43*E*+03	2.20*E*+02	5.21*E*+02	4.98*E*-02	6.34*E*+02	2.32*E*+00
SCA_PSO	4.77*E*+02	4.19*E*+01	5.21*E*+02	6.37*E*-02	6.29*E*+02	3.03*E*+00
CGSCA	1.63*E*+03	2.92*E*+02	5.21*E*+02	5.14*E*-02	6.34*E*+02	2.33*E*+00
GWO	7.02*E*+02	2.37*E*+02	5.21*E*+02	5.08*E*-02	6.13*E*+02	2.06*E*+00
MFO	1.34*E*+03	8.51*E*+02	5.20*E*+02	1.59*E*-01	6.24*E*+02	3.73*E*+00
BA	4.40*E*+02	3.98*E*+01	5.21*E*+02	5.19*E*-02	6.34*E*+02	3.36*E*+00
PSO	4.68*E*+02	3.39*E*+01	5.21*E*+02	4.82*E*-02	6.23*E*+02	2.99*E*+00
LSHADE	4.04*E*+02	1.61*E*+01	5.20*E*+02	1.00*E*-03	6.11*E*+02	2.23*E*+00

	F7		F8		F9	
	Avg	Std	Avg	Std	Avg	Std

ESCA_PSO	7.02*E*+02	5.88*E*-02	9.83*E*+02	2.14*E*+01	1.13*E*+03	2.09*E*+01
SCADE	9.10*E*+02	3.53*E*+01	1.07*E*+03	1.63*E*+01	1.21*E*+03	1.63*E*+01
SCA	8.43*E*+02	2.36*E*+01	1.04*E*+03	2.05*E*+01	1.18*E*+03	1.64*E*+01
SCA_PSO	7.01*E*+02	7.70*E*-02	9.97*E*+02	3.65*E*+01	1.13*E*+03	3.53*E*+01
CGSCA	8.67*E*+02	2.74*E*+01	1.06*E*+03	1.61*E*+01	1.18*E*+03	1.59*E*+01
GWO	7.23*E*+02	1.75*E*+01	8.81*E*+02	1.77*E*+01	9.99*E*+02	2.43*E*+01
MFO	8.15*E*+02	7.39*E*+01	9.36*E*+02	2.91*E*+01	1.12*E*+03	5.57*E*+01
BA	7.01*E*+02	1.55*E*-01	1.03*E*+03	4.75*E*+01	1.20*E*+03	6.92*E*+01
PSO	7.02*E*+02	1.62*E*-01	9.71*E*+02	2.31*E*+01	1.12*E*+03	3.57*E*+01
LSHADE	7.00*E*+02	1.17*E*-02	8.00*E*+02	1.82*E*-01	9.36*E*+02	1.36*E*+01

	F10		F11		F12	
	Avg	Std	Avg	Std	Avg	Std

ESCA_PSO	4.71*E*+03	6.56*E*+02	5.69*E*+03	6.28*E*+02	1.20*E*+03	3.92*E*-01
SCADE	7.41*E*+03	3.71*E*+02	8.10*E*+03	3.58*E*+02	1.20*E*+03	2.15*E*-01
SCA	6.93*E*+03	4.80*E*+02	8.10*E*+03	3.38*E*+02	1.20*E*+03	2.81*E*-01
SCA_PSO	5.26*E*+03	7.19*E*+02	5.62*E*+03	7.81*E*+02	1.20*E*+03	3.01*E*-01
CGSCA	7.19*E*+03	3.88*E*+02	8.05*E*+03	3.20*E*+02	1.20*E*+03	2.86*E*-01
GWO	3.34*E*+03	4.08*E*+02	3.93*E*+03	4.80*E*+02	1.20*E*+03	8.77*E*-01
MFO	4.56*E*+03	9.40*E*+02	5.40*E*+03	8.30*E*+02	1.20*E*+03	2.55*E*-01
BA	5.16*E*+03	6.27*E*+02	5.43*E*+03	6.13*E*+02	1.20*E*+03	3.10*E*-01
PSO	4.97*E*+03	5.63*E*+02	5.70*E*+03	5.81*E*+02	1.20*E*+03	2.82*E*-01
LSHADE	1.00E+03	7.66*E*-01	2.91*E*+03	4.12E+02	1.20*E+*03	3.80*E*-02

	F13		F14		F15	
	Avg	Std	Avg	Std	Avg	Std

ESCA_PSO	1.30*E*+03	9.71*E*-02	1.40*E*+03	3.81*E*-02	1.52*E*+03	1.41*E*+00
SCADE	1.30*E*+03	3.33*E*-01	1.49*E*+03	1.18*E*+01	2.17*E*+04	7.85*E*+03
SCA	1.30*E*+03	3.27*E*-01	1.45*E*+03	8.31*E*+00	5.16*E*+03	3.72*E*+03
SCA_PSO	1.30*E*+03	6.25*E*-02	1.40*E*+03	4.86*E*-02	1.52*E*+03	1.49*E*+00
CGSCA	1.30*E*+03	3.16*E*-01	1.45*E*+03	1.06*E*+01	8.10*E*+03	5.63*E*+03
GWO	1.30*E*+03	3.97*E*-01	1.41*E*+03	7.06*E*+00	1.82*E*+03	8.98*E*+02
MFO	1.30*E*+03	1.45*E*+00	1.43*E*+03	2.16*E*+01	1.28*E*+05	3.08*E*+05
BA	1.30*E*+03	1.38*E*-01	1.40*E*+03	4.97*E*-02	1.53*E*+03	6.26*E*+00
PSO	1.30*E*+03	7.09*E*-02	1.40*E*+03	1.19*E*-01	1.52*E*+03	1.11*E*+00
LSHADE	1.30*E*+03	7.43E-02	1.40*E*+03	9.17E-02	1.51*E*+03	1.76*E*+00

	F16		F17		F18	
	Avg	Std	Avg	Std	Avg	Std

ESCA_PSO	1.61*E*+03	3.67E-01	4.35*E*+05	2.41*E*+05	1.93*E*+06	6.44*E*+05
SCADE	1.61*E*+03	2.26*E*-01	1.58*E*+07	5.49*E*+06	1.54*E*+08	9.16*E*+07
SCA	1.61*E*+03	2.37*E*-01	5.52*E*+06	2.43*E*+06	1.74*E*+08	7.49*E*+07
SCA_PSO	1.61*E*+03	4.47*E*-01	1.79*E*+05	1.09*E*+05	7.62*E*+05	4.43*E*+05
CGSCA	1.61*E*+03	2.29*E*-01	6.77*E+*06	3.75*E*+06	1.43*E*+08	7.47*E*+07
GWO	1.61*E*+03	7.29*E*-01	1.49*E*+06	1.54*E*+06	2.88*E*+06	1.02*E*+07
MFO	1.61*E*+03	4.74*E*-01	2.40*E*+06	3.10*E*+06	2.64*E*+07	9.98*E*+07
BA	1.61*E*+03	2.59*E*-01	1.09*E*+05	8.01*E*+04	9.42*E*+04	4.63*E*+04
PSO	1.61E+03	5.31*E*-01	2.76*E*+05	1.21*E*+05	2.19*E*+06	7.43*E*+05
LSHADE	1.61*E*+03	3.85*E*-01	1.49*E*+04	6.33*E*+04	1.95*E*+03	5.46*E*+01

	F19		F20		F21	
	Avg	Std	Avg	Std	Avg	Std

ESCA_PSO	1.92*E*+03	2.29*E*+00	3.81*E*+03	1.57*E*+03	1.29*E*+05	1.10*E*+05
SCADE	2.02*E*+03	1.98*E*+01	2.52*E*+04	1.06*E*+04	2.18*E*+06	1.12*E*+06
SCA	1.99*E*+03	2.80*E*+01	1.56*E*+04	3.39*E*+03	1.23*E*+06	6.00*E*+05
SCA_PSO	1.92*E*+03	2.72*E*+00	2.47*E*+03	2.22*E*+02	9.35*E*+04	4.63*E*+04
CGSCA	1.99*E*+03	1.65*E*+01	1.88*E*+04	5.54*E*+03	1.67*E*+06	7.22*E*+05
GWO	1.94*E*+03	2.47*E*+01	1.97*E*+04	1.35*E*+04	6.56*E*+05	1.16*E*+06
MFO	1.96*E*+03	4.95*E*+01	7.19*E*+04	8.18*E*+04	8.20*E*+05	1.10*E*+06
BA	1.92*E*+03	1.83*E*+01	2.36*E*+03	1.13*E*+02	5.26*E+*04	3.10*E*+04
PSO	1.92*E*+03	2.43*E*+00	2.32*E*+03	7.07*E*+01	1.17*E*+05	6.92*E*+04
LSHADE	1.91*E*+03	1.84*E*+00	3.11*E*+03	3.51*E*+03	2.78*E*+03	2.77*E*+02

	F22		F23		F24	
	Avg	Std	Avg	Std	Avg	Std

ESCA_PSO	2.97*E*+03	2.43*E*+02	2.50*E*+03	0.00*E*+00	2.60*E*+03	0.00*E*+00
SCADE	3.11*E*+03	1.85*E*+02	2.50*E*+03	0.00*E*+00	2.60*E*+03	5.15*E*-06
SCA	2.99*E*+03	1.42*E*+02	2.67*E*+03	1.07*E*+01	2.60*E*+03	1.00*E*-01
SCA_PSO	3.17*E*+03	2.89*E*+02	2.50*E*+03	0.00*E*+00	2.60*E*+03	0.00*E*+00
CGSCA	3.07*E*+03	1.26*E*+02	2.50*E*+03	0.00*E*+00	2.60*E*+03	3.55*E*-06
GWO	2.59*E*+03	1.83*E*+02	2.63*E*+03	9.77*E*+00	2.60*E*+03	9.56*E*-04
MFO	3.12*E*+03	2.90*E*+02	2.66*E*+03	2.48*E*+01	2.68*E*+03	2.64*E*+01
BA	3.33*E*+03	3.17*E*+02	2.62*E*+03	3.12*E*-03	2.67*E*+03	3.46*E*+01
PSO	2.90*E*+03	2.61*E*+02	2.62*E*+03	7.09*E*-01	2.63*E*+03	5.18*E*+00
LSHADE	2.43*E*+03	9.48*E*+01	2.62*E*+03	1.88*E*-12	2.64*E*+03	6.32*E*+00

	F25		F26		F27	
	Avg	Std	Avg	Std	Avg	Std

ESCA_PSO	2.70*E*+03	0.00*E*+00	2.70*E*+03	1.27*E*-01	2.90*E*+03	0.00*E*+00
SCADE	2.70*E*+03	0.00*E*+00	2.70*E*+03	4.66*E*-01	3.20*E*+03	2.10*E*+02
SCA	2.73*E*+03	8.20*E*+00	2.70*E*+03	5.56*E*-01	3.57*E*+03	3.51*E*+02
SCA_PSO	2.70*E*+03	0.00*E*+00	2.77*E*+03	4.48*E*+01	2.90*E*+03	0.00*E*+00
CGSCA	2.70*E*+03	0.00*E*+00	2.70*E*+03	3.72*E*-01	2.90*E*+03	0.00*E*+00
GWO	2.71*E*+03	3.94*E*+00	2.74*E*+03	6.01*E*+01	3.32*E*+03	1.24*E*+02
MFO	2.72*E*+03	8.77*E*+00	2.70*E*+03	1.42*E*+00	3.66*E*+03	1.76*E*+02
BA	2.73*E*+03	1.44*E*+01	2.70*E*+03	1.35*E*-01	3.91*E*+03	4.20*E*+02
PSO	2.71*E*+03	5.98*E*+00	2.78*E*+03	4.07*E*+01	3.39*E*+03	2.97*E*+02
LSHADE	2.71*E*+03	3.23*E*+00	2.71*E*+03	3.04*E*+01	3.25*E*+03	9.56*E*+01

	F28		F29		F30	
	Avg	Std	Avg	Std	Avg	Std

ESCA_PSO	3.00*E*+03	0.00*E*+00	3.19*E*+03	8.63*E*+01	3.88*E*+03	6.83*E*+02
SCADE	4.96*E*+03	9.21*E*+02	1.91*E*+07	1.01*E*+07	4.90*E*+05	1.70*E*+05
SCA	4.84*E*+03	2.97*E*+02	1.37*E*+07	7.32*E*+06	2.39*E*+05	7.38*E*+04
SCA_PSO	3.00*E*+03	0.00*E*+00	1.26*E*+04	3.99*E*+04	1.53*E*+04	1.08*E*+04
CGSCA	3.00*E*+03	0.00*E*+00	3.10*E*+03	0.00*E*+00	3.20*E*+03	0.00*E*+00
GWO	3.84*E*+03	2.03*E*+02	6.26*E*+05	2.36*E*+06	4.88*E*+04	4.04*E*+04
MFO	3.98*E*+03	2.29*E*+02	3.06*E*+06	3.58*E*+06	5.65*E*+04	4.66*E*+04
BA	5.29*E*+03	6.59*E*+02	3.13*E*+07	3.38*E*+07	1.30*E*+04	1.23*E*+04
PSO	7.32*E*+03	8.69*E*+02	9.61*E*+04	1.83*E*+05	1.44*E*+04	7.29*E*+03
LSHADE	3.73*E*+03	7.27*E*+01	3.68*E*+03	4.12*E*+01	5.47*E*+03	1.26*E*+03

**(a):** 

*F*	ESCA_PSO	SCADE		SCA		SCA_PSO		CGSCA		GWO	
F1	N/A	1.73*E*-06	+	1.73*E*-06	+	2.80*E*-01		1.73*E*-06	+	2.88*E*-06	+
F2	N/A	1.73*E*-06	+	1.73*E*-06	+	1.73*E*-06	—	1.73*E*-06	+	1.73*E*-06	+
F3	N/A	1.73*E*-06	+	1.73*E*-06	+	1.92*E*-06	—	1.73*E*-06	+	1.73*E*-06	+
F4	N/A	1.73*E*-06	+	1.73*E*-06	+	8.77*E*-01		1.73*E*-06	+	1.92*E*-06	+
F5	N/A	1.78*E*-01		1.25*E*-02	—	6.27*E*-02		1.48*E*-02	—	1.59*E*-01	
F6	N/A	3.52*E*-06	+	1.02*E*-05	+	4.53*E*-01		1.24*E*-05	+	1.73*E*-06	—
F7	N/A	1.73*E*-06	+	1.73*E*-06	+	1.73*E*-06	—	1.73*E*-06	+	1.73*E*-06	+
F8	N/A	1.73*E*-06	+	1.92*E*-06	+	1.53*E*-01		1.73*E*-06	+	1.73*E*-06	—
F9	N/A	1.73*E*-06	+	2.35*E*-06	+	5.30*E*-01		1.73*E*-06	+	1.73*E*-06	—
F10	N/A	1.73*E*-06	+	1.73*E*-06	+	9.84*E*-03	+	1.73*E*-06	+	1.73*E*-06	—
F11	N/A	1.73*E*-06	+	1.73*E*-06	+	6.88*E*-01		1.73*E*-06	+	1.73*E*-06	—
F12	N/A	2.37*E*-05	+	2.58*E*-03	+	8.94*E*-01		4.53*E*-04	+	3.18*E*-01	
F13	N/A	1.73*E*-06	+	1.73*E*-06	+	4.99*E*-03	—	1.73*E*-06	+	2.43*E*-02	—
F14	N/A	1.73*E*-06	+	1.73*E*-06	+	2.70*E*-02	—	1.73*E*-06	+	5.22*E*-06	+
F15	N/A	1.73*E*-06	+	1.73*E*-06	+	5.44*E*-01		1.73*E*-06	+	4.86*E*-05	+
F16	N/A	3.88*E*-06	+	1.73*E*-06	+	1.96*E-*03	+	1.92*E*-06	+	2.88*E*-06	—
F17	N/A	1.73*E*-06	+	1.73*E*-06	+	1.48*E*-04	—	1.73*E*-06	+	7.71*E*-04	+
F18	N/A	1.73*E*-06	+	1.73*E*-06	+	2.35*E*-06	—	1.73*E*-06	+	2.07*E*-02	+
F19	N/A	1.73*E*-06	+	1.73*E*-06	+	7.97*E*-01		1.73*E*-06	+	1.74*E*-04	+
F20	N/A	1.73*E*-06	+	1.73*E*-06	+	1.92*E*-06	—	1.73*E*-06	+	2.88*E*-06	+
F21	N/A	1.73*E*-06	+	1.73*E*-06	+	7.19*E*-02		1.73*E*-06	+	1.15*E*-04	+
F22	N/A	6.42*E*-03	+	3.18*E*-01		4.11*E*-03	+	1.36*E*-01		7.69*E*-06	—
F23	N/A	1.00*E*+00		1.73*E*-06	+	1.00*E*+00		1.00*E*+00		1.73*E*-06	+
F24	N/A	1.56*E*-02	+	1.73*E*-06	+	1.00*E*+00		2.44*E*-04	+	1.73*E*-06	+
F25	N/A	1.00*E*+00		1.73*E*-06	+	1.00*E*+00		1.00*E*+00		3.79*E*-06	+
F26	N/A	1.73*E*-06	+	1.73*E*-06	+	1.64*E*-05	+	1.73*E*-06	+	4.68*E*-03	+
F27	N/A	5.96*E*-05	+	1.73*E*-06	+	1.00*E*+00		1.00*E*+00		1.73*E*-06	+
F28	N/A	1.23*E*-05	+	1.73*E*-06	+	1.00*E*+00		1.00*E*+00		1.73*E*-06	+
F29	N/A	1.73*E*-06	+	1.73*E*-06	+	5.11*E*-03	+	5.61*E*-06	—	1.73*E*-06	+
F30	N/A	1.73*E*-06	+	1.73*E*-06	+	6.75*E*-05	+	1.32*E*-04	—	1.73*E*-06	+
+/-/=	/	27/0/3		28/1/1		6/8/10		22/3/5		20/8/2	
Avg	2	10		9		3		7		5	

**(b):** 

*F*	MFO		BA		PSO		LSHADE	
F1	3.18*E*-06	+	1.73*E*-06	—	2.99*E*-01		1.73*E*-06	—
F2	1.73*E*-06	+	1.73*E*-06	—	1.73*E*-06	+	1.73*E*-06	—
F3	1.73*E*-06	+	1.73*E*-06	—	1.73*E*-06	—	1.73*E*-06	—
F4	1.73*E*-06	+	1.57*E*-02	—	9.75*E*-01		1.73*E*-06	—
F5	1.73*E*-06	—	8.45*E*-01		1.53*E*-01		1.73*E*-06	—
F6	1.15*E*-04	—	3.06*E*-04	+	7.69*E*-06	—	1.73*E*-06	—
F7	1.73*E*-06	+	1.73*E*-06	—	1.73*E*-06	+	1.73*E*-06	—
F8	1.64*E*-05	—	2.83*E*-04	+	5.45*E*-02		1.73*E*-06	—
F9	2.21*E*-01		7.51*E*-05	+	2.80*E*-01		1.73*E*-06	—
F10	4.53*E*-01		4.68*E*-03	+	1.85*E*-01		1.73*E*-06	—
F11	1.92*E*-01		1.11*E*-01		9.26*E*-01		1.73*E*-06	—
F12	1.73*E*-06	—	1.73*E*-06	—	4.20*E*-04	+	1.73*E*-06	—
F13	1.73*E*-06	+	6.56*E*-02		7.16*E*-04	—	1.80*E*-05	—
F14	1.73*E*-06	+	1.64*E*-05	+	1.48*E*-02	+	8.19*E*-05	+
F15	1.73*E*-06	+	1.92*E*-06	+	5.32*E*-03	—	1.73*E*-06	—
F16	4.29*E*-06	+	1.73E-06	+	5.30*E*-01		1.73*E*-06	—
F17	2.41*E*-03	+	2.88*E*-06	—	2.41*E*-03	—	2.13*E*-06	—
F18	3.59*E*-04	+	1.73*E*-06	—	1.85*E*-01		1.73*E*-06	—
F19	2.05*E*-04	+	6.87*E*-02		5.45*E*-02		1.73*E*-06	—
F20	1.73*E*-06	+	1.92*E*-06	—	1.92*E*-06	—	3.59*E*-04	—
F21	1.36*E*-04	+	2.84*E*-05	—	7.19*E*-01		1.73*E*-06	—
F22	4.72*E*-02	+	1.15*E*-04	+	2.21*E*-01		1.73*E*-06	—
F23	1.73*E*-06	+	1.73*E*-06	+	1.73*E*-06	+	4.32*E*-08	+
F24	1.73*E*-06	+	1.73*E*-06	+	1.73*E*-06	+	1.73*E*-06	+
F25	1.73*E*-06	+	1.73*E*-06	+	1.73*E*-06	+	1.73*E*-06	+
F26	1.73*E*-06	+	7.52*E*-02		1.24*E*-05	+	1.02*E*-01	
F27	1.73*E*-06	+	1.73*E*-06	+	1.73*E*-06	+	1.73*E*-06	+
F28	1.73*E*-06	+	1.73*E*-06	+	1.73*E*-06	+	1.73*E*-06	+
F29	1.73*E*-06	+	1.73*E*-06	+	8.73*E*-03	+	1.73*E*-06	+
F30	1.73*E*-06	+	1.73*E*-06	+	1.73*E*-06	+	4.29*E*-06	+
+/-/=	23/4/3		15/10/5		12/6/12		8/21/1	
Avg	8		6		4		1	

The article "Boosted Sine Cosine Algorithm with Application to Medical Diagnosis" was published in 2022. Journal: Comput Math Methods Med.

**Table 5:** Results of mutation mechanism comparison experiment.

	F1		F2		F3	
	Avg	Stdv	Avg	Stdv	Avg	Stdv

ESCA_PSO	1.0121*E*+07	4.1281*E*+06	7.2870*E*+07	6.7257*E*+06	9.0781*E*+03	1.6748*E*+03
ESCA_PSO1	1.0956*E*+07	6.3712*E*+06	7.5147*E*+07	7.5579*E*+06	9.4351*E*+03	2.5065*E*+03
ESCA_PSO2	8.8248*E*+06	4.3297*E*+06	7.5579*E*+07	6.4189*E*+06	8.9495*E*+03	2.0387*E*+03
ESCA_PSO3	8.9362*E*+06	3.2913*E*+06	7.6554*E*+07	5.5330*E*+06	8.2034*E*+03	2.8244*E*+03

	F4		F5		F6	
	Avg	Stdv	Avg	Stdv	Avg	Stdv

ESCA_PSO	4.7228*E*+02	4.7567*E*+01	5.2095*E*+02	7.3218*E*-02	6.2832*E*+02	3.6455*E*+00
ESCA_PSO1	4.8246*E*+02	4.3094*E*+01	5.2093*E*+02	5.9358*E*-02	6.2994*E*+02	3.6753*E*+00
ESCA_PSO2	4.8304*E*+02	3.1844*E*+01	5.2095*E*+02	4.0250*E*-02	6.2907*E*+02	2.8954*E*+00
ESCA_PSO3	4.6323*E*+02	3.5952*E*+01	5.2094*E*+02	6.0599*E*-02	6.2602*E*+02	3.6698*E*+00

	F7		F8		F9	
	Avg	Stdv	Avg	Stdv	Avg	Stdv

ESCA_PSO	7.0165*E*+02	6.6719*E*-02	9.7250*E*+02	1.7061*E*+01	1.1273*E*+03	2.1663*E*+01
ESCA_PSO1	7.0165*E*+02	5.8391*E*-02	9.7622*E*+02	2.0619*E*+01	1.1213*E*+03	2.3921*E*+01
ESCA_PSO2	7.0164*E*+02	4.8112*E*-02	9.7878*E*+02	1.5477*E*+01	1.1222*E*+03	2.4011*E*+01
ESCA_PSO3	7.0163*E*+02	6.2317*E*-02	9.5729*E*+02	1.6848*E*+01	1.1358*E*+03	3.5018*E*+01

	F10		F11		F12	
	Avg	Stdv	Avg	Stdv	Avg	Stdv

ESCA_PSO	4.9137*E*+03	7.2648*E*+02	5.6985*E*+03	5.0594*E*+02	1.2023*E*+03	3.2946*E*-01
ESCA_PSO1	4.9133*E*+03	6.5258*E*+02	5.6409*E*+03	7.1573*E*+02	1.2023*E*+03	2.7883*E*-01
ESCA_PSO2	4.9278*E*+03	6.4952*E*+02	5.6196*E*+03	5.2887*E*+02	1.2023*E*+03	2.8632*E*-01
ESCA_PSO3	3.9106*E*+03	7.0806*E*+02	5.7900*E*+03	6.4145*E*+02	1.2025*E*+03	1.9371*E*-01

	F13		F14		F15	
	Avg	Stdv	Avg	Stdv	Avg	Stdv

ESCA_PSO	1.3005*E*+03	8.0129*E*-02	1.4003*E*+03	5.5878*E*-02	1.5178*E*+03	1.8461*E*+00
ESCA_PSO1	1.3004*E*+03	6.5982*E*-02	1.4002*E*+03	3.9799*E*-02	1.5176*E*+03	1.4145*E*+00
ESCA_PSO2	1.3005*E*+03	1.3432*E*-01	1.4003*E*+03	5.0665*E*-02	1.5173*E*+03	1.5482*E*+00
ESCA_PSO3	1.3004*E*+03	9.2885*E*-02	1.4003*E*+03	1.0046*E*-01	1.5168*E*+03	1.2616*E*+00

	F16		F17		F18	
	Avg	Stdv	Avg	Stdv	Avg	Stdv

ESCA_PSO	1.6119*E*+03	3.7281*E*-01	3.5341*E*+05	1.5577*E*+05	1.9265*E*+06	5.4288*E*+05
ESCA_PSO1	1.6121*E*+03	2.7974*E*-01	4.7094*E*+05	5.3309*E*+05	1.9803*E*+06	5.1404*E*+05
ESCA_PSO2	1.6120*E*+03	3.9442*E*-01	4.2443*E*+05	3.0521*E*+05	2.1497*E*+06	4.0650*E*+05
ESCA_PSO3	1.6117*E*+03	3.5803*E*-01	4.4610*E*+05	3.0212*E*+05	1.7955*E*+06	4.8630*E*+05

	F19		F20		F21	
	Avg	Stdv	Avg	Stdv	Avg	Stdv

ESCA_PSO	1.9176*E*+03	2.6584*E*+00	4.6963*E*+03	2.1120*E*+03	1.5933*E*+05	1.2738*E*+05
ESCA_PSO1	1.9195*E*+03	1.1064*E*+01	4.8166*E*+03	2.4521*E*+03	1.6422*E*+05	1.1183*E*+05
ESCA_PSO2	1.9182*E*+03	2.6893*E*+00	4.2130*E*+03	1.8120*E*+03	1.7741*E*+05	1.5670*E*+05
ESCA_PSO3	1.9210*E*+03	1.6909*E*+01	2.5728*E*+03	3.9978*E*+02	1.2953*E*+05	9.6487*E*+04

	F22		F23		F24	
	Avg	Stdv	Avg	Stdv	Avg	Stdv

ESCA_PSO	3.0075*E*+03	2.5470*E*+02	2.5000*E*+03	0.0000*E*+00	2.6000*E*+03	0.0000*E*+00
ESCA_PSO1	3.0277*E*+03	1.8557*E*+02	2.5000*E*+03	0.0000*E*+00	2.6000*E*+03	0.0000*E*+00
ESCA_PSO2	2.9865*E*+03	2.5463*E*+02	2.5000*E*+03	0.0000*E*+00	2.6000*E*+03	0.0000*E*+00
ESCA_PSO3	2.8237*E*+03	2.0355*E*+02	2.5942*E*+03	4.7914*E*+01	2.6000*E*+03	3.1173*E*-04

	F25		F26		F27	
	Avg	Stdv	Avg	Stdv	Avg	Stdv

ESCA_PSO	2.7000*E*+03	0.0000*E*+00	2.7004*E*+03	7.7168*E*-02	2.9000*E*+03	0.0000*E*+00
ESCA_PSO1	2.7000*E*+03	0.0000*E*+00	2.7004*E*+03	9.2230*E*-02	2.9000*E*+03	0.0000*E*+00
ESCA_PSO2	2.7000*E*+03	0.0000*E*+00	2.7137*E*+03	3.4412*E*+01	2.9000*E*+03	0.0000*E*+00
ESCA_PSO3	2.7000*E*+03	0.0000*E*+00	2.7004*E*+03	7.1707*E*-02	3.4906*E*+03	3.4856*E*+02

	F28		F29		F30	
	Avg	Stdv	Avg	Stdv	Avg	Stdv

ESCA_PSO	3.0000*E*+03	0.0000*E*+00	3.1619*E*+03	5.6888*E*+01	3.7103*E*+03	6.0049*E*+02
ESCA_PSO1	3.0000*E*+03	0.0000*E*+00	3.4574*E*+03	4.0471*E*+02	5.0126*E*+03	1.8702*E*+03
ESCA_PSO2	3.0000*E*+03	0.0000*E*+00	7.4310*E*+04	2.6321*E*+05	1.1615*E*+04	8.8958*E*+03
ESCA_PSO3	3.9181*E*+03	8.8744*E*+02	3.1047*E*+03	4.4337*E*+00	3.2472*E*+03	4.9782*E*+01

The article "Boosted Sine Cosine Algorithm with Application to Medical Diagnosis" was published in 2022. Journal: Comput Math Methods Med.

**Table 6:** Results obtained by ESCA_PSO-SVM on the Bupa liver problem.

Fold	ACC (%)	Sensitivity (%)	Specificity (%)	MCC
No. 1	74.29	61.54	81.82	0.4414
No. 2	67.65	36.36	82.61	0.2092
No. 3	80.00	71.43	85.71	0.5794
No. 4	82.35	90.91	78.26	0.6517
No. 5	82.35	64.29	95.00	0.6404
No. 6	71.43	54.55	79.17	0.3371
No. 7	64.71	55.56	75.00	0.3099
No. 8	62.86	38.89	88.24	0.3102
No. 9	77.14	65.00	93.33	0.5893
No. 10	67.65	53.33	78.95	0.3354
Avg.	73.04	59.18	83.81	0.4404
Max	82.35	90.91	95.00	0.6517
Min	62.86	36.36	75.00	0.2092

**Table 7:** Results obtained by ESCA_PSO-SVM on the Cleveland heart problem.

Fold	ACC (%)	Sensitivity (%)	Specificity (%)	MCC
No. 1	76.67	72.22	83.33	0.5443
No. 2	87.10	78.57	94.12	0.7427
No. 3	83.33	76.92	88.24	0.6591
No. 4	77.42	76.92	77.78	0.5424
No. 5	80.00	69.23	88.24	0.5909
No. 6	76.67	78.57	75.00	0.5345
No. 7	83.33	87.50	78.57	0.6652
No. 8	83.33	50.00	100.00	0.6325
No. 9	93.55	90.00	95.24	0.8524
No. 10	86.67	88.89	83.33	0.7222
Avg.	82.81	76.88	86.38	0.6486
Max	93.55	90.00	100.00	0.8524
Min	76.67	50.00	75.00	0.5345

## Data Availability

The data involved in this study are all public data, which can be downloaded through public channels.
